# The lncRNA XIST promotes colorectal cancer cell growth through regulating the miR-497-5p/FOXK1 axis

**DOI:** 10.1186/s12935-020-01647-4

**Published:** 2020-12-10

**Authors:** Nan Wang, Jia-Xing He, Guo-Zhan Jia, Ke Wang, Shuai Zhou, Tao Wu, Xian-Li He

**Affiliations:** Department of General Surgery, Tangdu Hospital, the Air Force Medical University, 710038 Xi’an, China

**Keywords:** LncRNA XIST, miR-497-5p, FOXK1, Colon cancer cell carcinoma

## Abstract

**Background:**

Recent studies suggest that long noncoding RNAs (lncRNAs) play an important role in tumorigenesis. As a newly identified lncRNA, the role of XIST in colorectal cancer (CRC) has not been established. Here, we sought to characterize the role of XIST and its associated regulatory network in CRC cells.

**Methods:**

Expression of XIST mRNA, miR-497-5p, and forkhead box k1 (FOXK1) in CRC cells and tissues were detected using quantitative real-time polymerase chain reaction (qRT-PCR). Proliferation and apoptosis of CRC cells were determined using the CCK-8 cell counting assay and flow cytometry. The rate of cell migration and invasion was determined using a transwell assay. The relationships between XIST, miR-497-5p, and FOXK1 were predicted and confirmed using a dual-luciferase reporter assay. Expression of FOXK1 protein was quantified by Western blot.

**Results:**

XIST and FOXK1 expression were significantly upregulated in CRC tissues and cell lines, while miR-497-5p expression was downregulated. XIST knockdown significantly suppressed CRC cell proliferation, migration, and invasion. Silencing of XIST also reversed the downregulation of miR-497-5p and upregulation of FOXK1. Moreover, blocking XIST expression was shown to inhibit CRC tumor growth *in vivo* and the effects were antagonized by the loss of miR-497-5p. miR-497-5p was shown to act as a sponge of XIST and also targeted FOXK1 in CRC cells.

**Conclusions:**

XIST was shown to promote the malignancy of CRC cells by competitively binding to miR-497-5p, resulting in an increase in FOXK1 expression. These results suggest that targeting of XIST may represent a possible treatment for CRC.

## Background

Colorectal cancer (CRC) is a common malignancy, accounting for 9.2% of all cancers [1], with lower incidence seen in developed countries, relative to those with less developed economies [2]. Despite substantial progress in surgical techniques and other anti-cancer treatments, treatment outcomes for CRC have not significantly improved. Surgery remains the only proven curative treatment for CRC; however, such treatments are not possible for the majority of patients with advanced CRC [3]. The development of new treatment options is therefore urgently needed to address these unmet needs [4]. To achieve these goals, we will need a better understanding of the molecular mechanisms underlying CRC pathogenesis to improve both the diagnosis and treatment of CRC.

Long non-coding RNAs (lncRNAs) are a newly discovered class of RNA molecules that are typically over 200 nt in length. LncRNAs have been shown to play a role in a wide variety of cellular functions including cell differentiation, development, apoptosis, proliferation, and metabolism [5]. X-inactivation-specific transcript (XIST), a novel lncRNA located at the X-inactivation center, may alter heterochromatin stability leading to changes in gene expression, thereby affecting cancer progression [6]. It has been reported that XIST overexpression is highly correlated with poorer prognoses in patients with various cancers, including colon cancer [7], pancreatic cancer [8], and brain cancer [9]; however, the role of XIST in CRC remains poorly understood.

MicroRNAs (miRNAs), approximately 22 nucleotides in length, have been shown to confer a wide range of activities by targeting gene expression at the post-transcriptional level [10]. As miRNAs help to regulate a wide array of cellular processes including metabolism, differentiation, and apoptosis, any dysregulation of these transcripts may contribute to disease pathology [11, 12]. Among the various miRNAs described to date, miR-497-5p has been identified as a promising therapeutic target for CRC [13]. Similarly, the forkhead box protein FOXK1 has also been shown to contribute to the incidence, progression, invasion, and metastasis of various tumors such as esophageal cancer [14], glioma [15], colon cancer [16], and gastric cancer [17].

In the present study, we performed as series of *in vitro* and *in vivo* experiments to understand more fully the various activities of XIST in CRC, providing new insights into the potential mechanism of action of XIST in CRC.

## Methods

### Sample collection

Fifty-four paired CRC tissues and adjacent non-tumor tissues were collected from March 2015 to May 2019 in Tangdu Hospital, the Air Force Medical University, Xi’an, China. Informed consent was obtained from all patients or their guardians and the study was approved by the Ethics Committee of our institution.

### Cell culture and transfection

Four CRC cell lines (including LOVO, SW480, HT-29, and HCT-116) and one normal colon epithelial cell line (FHC) were obtained from Shanghai Institute of Biochemistry and Cell Biology (Shanghai, China). All cell lines were cultured in DMEM (Gibco, USA) supplemented with 10% fetal bovine serum (FBS; Tianhang, Hangzhou, China) and 1% penicillin-streptomycin in a humidified incubator (37 °C, 5% CO_2_). Small interfering RNA targeting XIST (si-XIST: 5′-GCCCUUCUCUUCGAACUGUTT-3′) and its matching control (si-NC: 5′-CGTTAATCGCGTATAATACGCGTAT-3′), were obtained from Genepharma (Shanghai, China). A miR-497-5p mimic (miR-497-5p), its inhibitor (anti-miR-497-5p), and their corresponding controls (miR-NC and anti-miR-NC) were obtained from Ribobio (Guangzhou, China). For overexpression vectors, the sequence of FOXK1 was cloned into the pcDNA3.1 vector (vector) according to the manufacturer’s instructions (Life Technologies). Briefly, 100 nM of miR-497-5p mimics or miR-497-5p inhibitor and 1000 ng plasmid were transfected into each 6-well plate for 48 h using Lipofectamine 3000 (Invitrogen, Waltham, MA, USA). For animal experiments, cells were stably transfected with an XIST lentiviral vector, constructed by Hanyin Biotechnology Co., Ltd., Shanghai, China. After transfection, DMEM medium was replaced with DMEM supplemented with puromycin (3 µg/mL) as a positive selection for infected cells.

### Cell proliferation assays

The viability of HT29 and SW480 cells was evaluated using the Cell Counting Kit-8 assay (CCK-8, Dojindo, Kumamoto, Japan). HT29 and SW480 cells (1 × 10^3^cells/mL per 96-well plate) were cultured for 24, 48, and 72 h, respectively. For the cell proliferation assay, each well was treated with 10 µL CCK-8 solution for 2 h. Absorbance was detected at 450 nm using a standard microplate reader.

### Flow cytometric analysis of apoptosis

HT29 and SW480 cells were harvested and fixed in pre-cooled ethanol, then resuspended in cold buffer containing 5 µL Annexin V-FITC. The samples were treated with 5 µL PI and 200 µL binding buffer and incubated for 5 min. Cell apoptosis was then analyzed using an Annexin FITC/PI flow cytometry assay kit.

### Cell migration and invasion assay

A transwell assay was used to assess cell migration and invasion. The upper chamber was coated with Matrigel (8.0 µm PET membrane, 24 well plate, Corning, USA), after which cells were added at a density of 1 × 10^4^ cells/well and cultured in 400 µL serum-free DMEM medium. Next, 600 µL DMEM supplemented with 10% FBS was added to the lower chamber. Cells were then incubated for 24 h, after which cells on the bottom of the upper chamber were fixed with 90% ethanol solution for 30 min. Cells were then stained with 0.1% crystal violet for 10 min, and the degree of invasion was observed using a light microscope (Olympus, Japan).

### Dual-luciferase reporter assay

XIST or FOXK1 sequences containing a miR-497-5p binding site were amplified by PCR and cloned to a psiCHECK-2 vector (Promega, Madison, WI, USA) to generate XIST-WT (wild-type) or FOXK1-WT (wild-type). The binding site of XIST was mutated to obtain the XIST-MUT (mutant type) or FOXK1-MUT (mutant type) using a Site-Directed Mutagenesis Kit (Stratagene, California, USA). XIST-WT, XIST-MUT, FOXK1-WT, and FOXK1-MUT were then co-transfected along with a miR-497-5p mimic into HT-29 and SW480 cells. Luciferase activities were detected using a dual-luciferase reporter assay system (Promega, Madison, USA).

### RNA isolation and quantitative reverse transcription polymerase (qRT-PCR)

Total RNA extraction was conducted using Trizol Reagent (Shanghai Pufei Biotech Co., Ltd., Shanghai, China). Reverse transcription into cDNA was conducted with Prime Script RT Master Mix (Takara Biotechnology Co., Ltd.) according to the manufacturer’s protocol. cDNA was obtained by reverse transcription after DNA elimination and amplified using SYBR Green Master Mixture (Takara, Otsu, Japan). The primer sequences are: LncRNA XIST: F: (5’-3’) AGC TCC TCG GAC AGC TGT AA; R: (5’-3’) CTC CAG ATA GCT GGC AAC C. miR-497-5p: F: (5’-3’) CCT TCA GCA GCA CAC TGT GG; R: (5’-3’) CAG TGC AGG GTC CGA GGT AT. FOXK1: F: (5’-3’) ACA CGT CTG GAG GAG ACA GC; R: (5’-3’) GAG AGG TTG TGC CGG ATA GA. GAPDH: F: (5’-3’) AAC GGA TTT GGT CGT ATT G; R: (5’-3’) GGA AGA TGG TGA TGG GAT T. The thermocycling conditions were applied as follows: denaturation at 95 °C for 5 min followed by 40 cycles at 95 °C for 30 sec, primer annealing at 60 °C for 30 sec, and primer extension at 72 °C for 5 min. Thermal cycling and real-time detection were conducted on a LightCycler 480 real-time PCR system (Roche, Indianapolis, Ind). The mRNA levels were calculated using the comparative (2^−△△Ct^) method.

### Western blot

Samples were lysed in RIPA buffer containing protease inhibitors. Total protein was isolated from cell or tissue lysates after centrifugation. The concentration of protein was assessed using a Bradford Protein Assay Kit (Beyotime, China). After quantification, 30 µg protein was resolved by SDS-PAGE and electro-transferred onto a polyvinylidene fluoride (PVDF) membrane (Millipore, Boston, MA, USA) (250 mA, 2 h), blocked with 5% skim milk for 1 h, and then incubated with primary antibodies anti-FOXK1 (1: 1000 dilution) or anti-β-actin (1: 5000 dilution, Cell Signaling Technology, USA) at 4 °C overnight, followed by incubation with appropriate secondary antibodies at room temperature for 1 h. Signal was detected using the enhanced chemiluminescence system.

### Xenograft tumor Model

Male BALB/c nude mice (~ 4 weeks of age) were purchased from Charles River (Beijing, China) and further used for the xenograft assays. All animal procedures were approved by the Ethics Committee for Animal Studies of Tangdu Hospital, the Air Force Medical University. HT29 cells (2 × 10^6^) transfected with si-XIST or si-NC were injected subcutaneously into one flank of each mouse. Total tumor volume was measured every four days. All mice were sacrificed after 24 days, and tumor masses were weighed and used for subsequent molecular analysis.

### Statistical analysis

All data of this study were expressed as the mean ± standard deviation (SD). SPSS 22.0 software was used to conduct all statistical analyses (SPSS, Inc, USA). The comparison between the data of the groups was analyzed by the Student’s t-test and two-way analysis of variance. The p-vale < 0.05 indicated statistical significance.

## Results

### XIST expression was upregulated in CRC tissues and cell lines

qPCR was used to measure XIST expression in CRC tissues and cells. XIST expression was shown to be significantly upregulated in CRC tissues relative to adjacent normal tissues (Fig. 1a, p *<* 0.01). Similarly, all CRC cell lines showed higher XIST expression compared to the FHC normal colon epithelial cell line (*p <* 0.01; Fig. 1b). Together, these results suggest that XIST is an oncogene in CRC.

**Fig. 1:** XIST expression is upregulated in CRC tissues and cell lines. **a** XIST expression in CRC tissues and matched normal tissues were determined using qRT-PCR. (**b**) XIST expression in CRC cell lines (HT29, HT116, SW480, and LOVO) and a normal colon epithelial cell line (FHC) were also determined using qRT-PCR. ^**^p < 0.01

### Inhibition of XIST expression attenuates cell malignancy in CRC cells

To determine further the role of XIST in CRC cells, the interference efficacy of si-XIST in HT29 and SW480 cells was confirmed by RT-qPCR (Fig. 2a). The CCK8 assay revealed significant inhibition of cell proliferation in HT29 and SW480 cells transfected with si-XIST (Fig. 2b), while flow cytometry revealed dramatic increases in apoptosis in si-XIST treated cells (Fig. 2c). In addition, the migration and invasive ability of HT29 and SW480 cells transfected with si-XIST were significantly decreased (Fig. 2d, e).

**Fig. 2:** Suppression of XIST expression reduced cell proliferation, migration, and invasion, and induced apoptosis in CRC cells. si-NC or si-XIST were transfected into HT29 and SW480 cells. Cell proliferation was measured using the CCK-8 assay (**a**) and flow cytometry was used to detect cell apoptosis (**b**). A transwell assay was used to measure the migration (**c**) and invasion (**d**) of cells. ^*^p < 0.05; ^**^p < 0.01

### XIST acts as a sponge for miR-497-5p in CRC

The relation between miR-497-5p and XIST was explored using the StarBase v2.0 online database. Sequence analysis indicated that XIST contains a potential binding site for miR-497-5p (Fig. 3a). A luciferase reporter gene assay revealed a significant decrease in luciferase activity of XIST-WT in CRC cells transfected with miR-497-5p mimic, but not in the XIST-MUT reporter (Fig. 3b). Moreover, miR-497-5p expression was significantly decreased in the CRC tissues (Fig. 3c) and cells (Fig. 3d). Silencing of XIST expression was shown to increase miR-497-5p levels significantly, while overexpression of miR-497-5p suppressed the levels of XIST (Fig. 3e and f).

**Fig. 3:** XIST acts as a sponge for miR-497-5p in CRC cells **a** Predicted binding sites between XIST and miR-497-5p are shown. **b** Luciferase activity was measured using a dual-luciferase reporter assay in cells co-transfected with pGL3-XIST-WT or pGL3-XIST-MUT vectors and miR-NC or miR-497-5p. **c**, **d** The expression of miR-497-5p was measured by qRT-PCR in CRC tissues and cell lines. **e** The expression of miR-497-5p was examined using qRT-PCR in HT29 and SW480 cells after transfection with si-XIST or si-NC. **f** XIST expression levels were determined in HT29 and SW480 cells after transfection with miR-497-5p or miRNA mimic. ^*^p < 0.05; ^**^p < 0.01

### Downregulation of miR-497-5p abolished si-XIST-mediated repression of CRC cells

Proliferation of HT29 and SW480 cells transfected with si-XIST was significantly inhibited compared with the negative control (Fig. 4a). Similarly, knockdown of miR-497-5p coupled with XIST downregulation attenuated the si-XIST-mediated arrest of cell proliferation. Flow cytometry analyses suggested that miR-497-5p inhibition significantly attenuated apoptosis promoted by XIST downregulation in HT29 and SW480 cells (Fig. 4b). Suppression of XIST significantly attenuated migration and invasion of HT29 and SW480 cells; however, these effects could be reversed following treatment with a miR-497-5p inhibitor (Fig. 4c, d).

**Fig. 4:** XIST inhibition affects cell behavior in CRC by acting as a sponge for miR-497-5p *in vitro*. HT29 and SW480 cells transfected with si-NC, si-XIST, si-XIST + miR-inhibitor NC, or si-XIST + miR-497-5p inhibitor were classified into four groups. **a** Cell proliferation was analyzed by CCK8 assay. **b** Flow cytometry was used to measure cell apoptosis. **c, d** A transwell assay was used to assess cell migration and invasion abilities. *p < 0.05; **p < 0.01

### The FOXK1 oncogene was suppressed by miR-497-5p

The TargetScan Human 7.2 online database predicted potential interactions between miR-497-5p and FOXK1 within the 3’UTR of FOXK1 (Fig. 5a). Luciferase assays revealed that miR-497-5p overexpression notably decreased the luciferase activities of FOXK1-WT and FOXK1-MUT, whereas the luciferase activity in FOXK1-MUT was unchanged (Fig. 5b**)**. Moreover, we observed a significant upregulation of FOXK1 mRNA (Fig. 5c**)** and protein expression (Fig. 5d**)** in CRC tissues and cell lines compared with normal controls (Fig. 5e). Furthermore, FOXK1 protein expression was determined to be markedly inhibited after miR-497-5p overexpression, which was restored by overexpression of XIST in HT29 and SW480 cells (Fig. 5f), suggesting that XIST could regulate FOXK1 via directly acting on miR-497-5p in CRC cells.

**Fig. 5:** FOXK1 is a target of miR-497-5p in CRC cells. **a** Predicted binding sites between FOXK1 and miR-497-5p are shown. **b** The luciferase activity was analyzed in HT29 and SW480 cells co-transfected with FOXK1-WT or FOXK1-MUT along with a miR-497-5p or NC mimic. **c, d** FOXK1 mRNA and protein expression were measured in CRC tissues and paired normal tissues by qRT-PCR or Western blot, respectively. **e** Expression of FOXK1 in HT29, SW480, FHC cells was measured by Western blot. **f** FOXK1 expression in HT29 and SW480 cells transfected with NC mimic, miR-497-5p, miR-497-5p + pcDNA, miR-497-5p + FOXK1 was detected by Western blot. ^*^p < 0.05; ^**^p < 0.01

### FOXK1 overexpression reversed miR-497-5p-mediated effects on CRC cells

Next, we sought to assess the regulatory effects of miR-497-5p on FOXK1. FOXK1 protein expression was significantly inhibited by XIST silencing in HT29 and SW480 cells (Fig. 6a). Moreover, silencing of XIST significantly inhibited cell proliferation (Fig. 6b) and was accompanied by a large increase in cell apoptosis (Fig. 6c). Interestingly, these effects may be partially inhibited via the overexpression of FOXK1 in HT29 and SW480 cells. Furthermore, cell migration and invasion were suppressed in the si-XIST group, but the opposite result was observed in the si-XIST + FOXK1 group, as determined using the Transwell assay (Fig. 6d, e). Together, these results indicate that FOXK1 may promote the progression of colon cancer cells and that FOXK1 binds directly to miR-497-5p.

**Fig. 6:** XIST silencing suppresses CRC progression via regulation of FOXK1 *in vitro*. HT29 and SW480 cells were transfected with si-NC, si-XIST, si-XIST + pcDNA, or si-XIST + FOXK1. **a** Expression of FOXK1 protein was measured by Western blot. **b** Cell proliferation was analyzed by CCK8 assay. **c** Cell apoptosis was analyzed using flow cytometry. **d, e** A transwell assay was used to assess cell migration and invasion abilities. ^*^p < 0.05; ^**^p < 0.01

### XIST deletion inhibits tumor growth in vivo

To determine the role of XIST for CRC *in vivo*, we established a xenograft model with SW480 cells stably transfected with si-XIST. As shown in Fig. 7a, compared with the si-NC group, both tumor volume and tumor weight were markedly decreased in the si-XIST group (Fig. 7b). Furthermore, qRT-PCR analyses showed that XIST and FOXK1 expression was notably decreased while miR-497-5p expression was significantly increased in the si-XIST group (Fig. 7c).

**Fig. 7:** Cells stably transfected with si-XIST were used to establish xenograft models. **a** Tumor volume was calculated every 4 days. **b** Mice were sacrificed, and tumor weight was examined in each group. **c** Expression of XIST, miR-497-5p and FOXK1 were detected in each groups by qRT-PCR. ^*^p < 0.05

## Discussion

A number of studies have shown strong associations between lncRNA expression and the occurrence and development of CRC. World epidemiological studies have found that African Americans have a higher incidence of colorectal cancer (CRC), and the fatality rate is higher than that of other populations. Using whole-genome sequencing technology, it is found that African Americans have more aberrations on chromosomes 11, 17 and X than whites, and the lncRNA XIST is the product of the X chromosome during the transcription process, suggesting that XIST may play an important role in the occurrence and prognosis of colorectal cancer[18]. ZHANG et al. [19] detected the expression of XIST in 196 clinical rectal cancer specimens and rectal cancer cell lines. Combined with the analysis of clinicopathological characteristics, it is found that the expression of lncRNA XIST is up-regulated in CRC cell lines and tissues, and the high expression of XIST is not only related to the tumor size, lymph node metastasis (TNM), distant metastasis and clinical stage of colorectal cancer, but also predicts shorter progression-free survival and overall survival in CRC patients. High expression of XIST has been confirmed as an independent risk factor for poor prognosis. Related luciferase binding experiments indicate that lncRNA XIST may achieve tumor migration and invasion of CRC by regulating the miR-137/EZH2 axis [20]. The lncRNA XIST/miR-486-5p/NRP-2 axis promotes the viability and epithelial-mesenchymal transition of CRC cells, thereby promoting the proliferation and inhibition of apoptosis of CRC cells [21]. XIST/miR-132-3p/MAPK1 axis promotes CRC cell proliferation by influencing the cell cycle [22]. The lncRNA XIST/miR-200b-3p/ZEB1 axis promotes the epithelial-mesenchymal transition (EMT) of CRC cells and the formation of CRC stem cells to regulate the growth and metastasis of CRC [23]. What’s more, XIST expression is up-regulated in drug-resistant CRC tissues and cells. Down-regulation of miR-124 expression or silencing of XIST can inhibit the negative regulation of SGK1 by miR-124, thereby reducing the IC50 value of doxorubicin, reducing P-gp and GST-π levels, enhancing cell apoptosis, and enhancing the drug sensitivity of doxorubicin, which provides new ideas for the study of drug resistance treatment strategies for CRC patients [24].

As a target of XIST, miR-497-5p was minimally expressed in CRC tissues and cells. However, when si-XIST was transfected into CRC cells, it led to an increase in miR-497-5p expression, thereby arresting colon cancer growth and metastasis. Conversely, the loss of miR-497-5p expression abolished the anti-cancer effects induced by the loss of XIST, indicating that XIST promotes CRC progression by directly affecting miR-497-5p expression.

FOXK1 plays a pivotal role in the etiology of many cancers [25]. Elevated expression of FOXK1 has been observed in breast cancer, and may contribute to pathogenesis by promoting cell proliferation and migration [26]. Increased FOXK1 expression has also been reported in gastric cancer tissues, as well as contributing to the invasion and metastasis of pancreatic cancer [27]. In this study, hsa-miR-497-5p was predicted to bind the 3’-UTR of FOXK1, resulting in weak expression of FOXK1 in colon cancer cells following upregulation of hsa-miR-497-5p. Notably, FOXK1 was highly expressed in CRC cells and tissues. Furthermore, the results of our rescue experiments revealed that the upregulation of FOXK1 reversed the inhibitory effect of miR-497-5p overexpression on proliferation, anti-apoptosis activity, and metastasis in CRC cells. Mechanistically, FOXK1 expression was upregulated in cells treated with si-XIST, with similar effects seen following the loss of miR-497-5p. Thus, our results showed that silencing XIST resulted in the downregulation of FOXK1 expression as XIST normally serves as a sponge for miR-497-5p in CRC cells. Subsequent *in vivo* experiments will be necessary to confirm these results.

## Conclusions

Both XIST (a lncRNA) and FOXK1 are overexpressed, while miR-497-5p is suppressed in CRC tissues and cells. Inhibition of XIST decreased cell growth, cell metastasis, and anti-apoptosis activity. Both XIST and FOXK1 were found to contain binding sites for miR-497-5p, as initially predicted in our study. Decreasing XIST expression was accompanied by an increase in miR-497-5p levels, while the upregulation of miR-497-5p produced similar inhibitory effects on CRC cells as that mediated by the loss of XIST. Mechanism studies confirmed that miR-497-5p negatively regulates FOXK1 and reverses FOXK1 expression induced by XIST in CRC cells. These observations may offer a promising strategy for the treatment of CRC.

## Data Availability

The data used to support the findings of this study are included in the article.

## Abbreviations

lncRNAs: Long noncoding RNAs
XIST: lncRNA XIST
CRC: Colorectal cancer
FOXK1: Forkhead box k1
qRT-PCR: Quantitative real-time polymerase chain reaction;
miRNAs: MicroRNAs
